# Neuroprotective Effect of Protein Phosphatase 2A/Tristetraprolin Following Subarachnoid Hemorrhage in Rats

**DOI:** 10.3389/fnins.2018.00096

**Published:** 2018-02-27

**Authors:** Jian Yin, Ran Li, Wenchao Liu, Yunchang Chen, Xin Zhang, Xifeng Li, Xuying He, Chuanzhi Duan

**Affiliations:** ^1^The National Key Clinic Specialty, The Neurosurgery Institute of Guangdong Province, Guangdong Provincial Key Laboratory on Brain Function Repair and Regeneration, Department of Neurosurgery, Zhujiang Hospital, Southern Medical University, Guangzhou, China; ^2^Departments of Neurosurgery, Hanghzou Red Cross Hospital, Hangzhou, China

**Keywords:** subarachnoid hemorrhage, early brain injury, protein phosphatase 2A, tristetraprolin, neuroinflammation, apoptosis

## Abstract

Early brain injury (EBI) following subarachnoid hemorrhage (SAH) can lead to inflammation and neuronal dysfunction. There is a need for effective strategies to mitigate these effects and improve the outcome of patients who experience SAH. The mRNA-destabilizing protein tristetraprolin (TTP) is an anti-inflammatory factor that induces the decay of cytokine transcripts and has been implicated in diseases such as glioma. However, the mechanism of action of TTP in EBI after SAH is unclear. The present study investigated the effects of TTP regulation via phosphorylation in a rat model of SAH by protein phosphatase (PP)2A, which is a pleiotropic enzyme complex with multiple substrate phospho-proteins. We hypothesized that inhibitory phosphorylation of TTP by PP2A would reduce neuroinflammation and apoptosis. To evaluate the function of each factor, the PP2A agonist FTY720, short interfering (si)RNAs targeting TTP and PP2A were administered to rats by intracerebroventricular injection 24 h before SAH. Rats were evaluated with SAH grade, neurological score, brain water content and by western blotting, and terminal deoxynucleotidyltransferase dUTP nick-end labeling. We found that endogenous PP2A and TTP levels were increased after SAH. FTY720 induced PP2A activation would lead to dephosphorylation and activation of TTP and decreased production of tumor necrosis factor (TNF)-α, interleukin (IL)-6, and IL-8. SiRNA-mediated TTP knockdown abolished anti-inflammatory effects of FTY720 treatment, indicating that PP2A was associated with TTP activation *in vivo*. Decreased TNF-α, IL-6, and IL-8 levels were associated with improvement of neurological function, reduction of brain edema, suppression of caspase-3, and up-regulation of B cell lymphoma-2. These results demonstrated that PP2A activation could enhance the anti-inflammatory and anti-apoptotic effects of TTP, by which it might shed light on the development of an effective therapeutic strategy against EBI following SAH.

## Introduction

Subarachnoid hemorrhage (SAH) is an acute cerebrovascular event that can have devastating consequences including disability and mortality (Chen et al., 2014). Early brain injury (EBI) typically occurs within 72 h after SAH and accounts for 60% of deaths as a result of increased intracranial pressure, reduced cerebral blood flow, and oxygen, oxidative stress, blood–brain barrier disruption, brain edema, inflammation, and neuronal apoptosis (Connolly et al., 2012; Sehba et al., 2012; Fujii et al., 2013). It has been proposed that suppressing inflammation and apoptosis can alleviate EBI after SAH.

Studies in rats have shown that inflammation and neuronal dysfunction are two important aspects of EBI following SAH (Guo et al., 2016; Yin et al., 2017). Levels of pro-inflammatory cytokines such as tumor necrosis factor (TNF)-α, interleukin (IL)-6, and IL-8 are increased after SAH. These factors can activate microglia and increase inflammatory cell infiltration into the brain, causing neuronal dysfunction (Chang et al., 2015; Niwa et al., 2016; Wu et al., 2016). Expression of these inflammation-related proteins may be affected by means of RNA-binding proteins, which could regulate mRNA stability by binding to AU-rich elements (AREs) in the 3′ untranslated region of transcripts and therefore counter the increase of cytokine levels (Hollams et al., 2002; Stoecklin and Anderson, 2006). This mechanism might be used as a therapeutic approach for preventing EBI after SAH.

Tristetraprolin (TTP) is a well-characterized RNA-binding protein that contains two zinc fingers necessary for ARE binding (Brooks and Blackshear, 2013) and inhibition of pro-inflammatory cytokine expression (e.g., TNF-α; IL-2, IL-6, IL-8, IL-10, and interferon γ) (Rachel et al., 2005; Sun et al., 2007; Suswam et al., 2008; Ogilvie et al., 2009; Schaljo et al., 2009). TTP has been reported to play a key role in the production of TNF-α, IL-6, and IL-8, whose transcripts contain AREs and therefore are targets of TTP-induced mRNA degradation (Sun et al., 2007; Rahman et al., 2016). As a result, TTP may suppress inflammation in EBI after SAH.

TTP has been implicated in many central nervous system disorders, including malignant glioma and brain ischemia (Jamison et al., 2008; Suswam et al., 2008). However, there were no reports to date regarding TTP expression in the brain and its role in SAH. Unphosphorylation increases the unstability of TTP and enhances its ability to ARE-containing decay (Rahman et al., 2015). Some studies have revealed that TTP is regulated by p38 mitogen-activated protein kinase (MAPK). However, inhibiting the latter does not increase the level of unphosphorylated TTP (Mahtani et al., 2001; Ross et al., 2017). Protein phosphatase (PP)2A activates TTP via dephosphorylation at S52 and S178, leading to the destabilization of target mRNAs (Marchese et al., 2010). Both PP2A and its agonist FTY720 have neuroprotective capacities against neuronal apoptosis in traumatic brain injury, acute ischemia, and neurodegenerative disease (Cipriani et al., 2015; Majd et al., 2016; Sangodkar et al., 2016; Tan et al., 2016). PP2A acts upstream of TTP signaling *in vitro* and *in vivo* (Rahman et al., 2016; Ross et al., 2017). The anti-inflammatory effects of TTP in brain tumors are generated through inhibiting TNF-α-induced expression of IL-8 and vascular endothelial growth factor and preventing its consequent neurovascular damage (Suswam et al., 2008). However, it is still unknown whether TTP can prevent EBI and improve brain function after SAH.

In this study, we speculated that TTP can attenuate neuronal inflammation and apoptosis associated with EBI following SAH. To test this hypothesis, we investigated the temporal expression profiles of PP2A and TTP in a rat model of SAH. And short interfering (si)RNA was used to knock down both factors on order to evaluate their effects on neurological functions and roles on neuroinflammation. We also assessed the anti-inflammatory and anti-apoptotic effects of the PP2A agonist FTY720 in the SAH model.

## Materials and methods

### Animals

Male Sprague-Dawley male rats weighing 280–320 g were purchased from the Animal Experiment Center of Southern Medical University (Guangzhou, China). Experimental and animal care procedures were approved by the Southern Medical University Ethics Committee.

### SAH model

The rat model of SAH was generated as previously described (Xie et al., 2017), with some modifications. Briefly, animals were anesthetized with 3% isoflurane in 60/40% medical air/oxygen. Rectal temperature was monitored and body temperature was maintained at approximately 37°C with an electric heating pad. The external carotid artery was identified and transected as a 3.0-mm stump. A sharpened 4–0 monofilament nylon suture was advanced rostrally into the internal carotid artery from the left external carotid artery stump until there was resistance, and then pushed 2.5 mm further into the bifurcation of the anterior and middle cerebral arteries until resistance was encountered. Immediately after puncture, the filament was withdrawn into the external carotid stump, and the internal carotid artery was reperfused to induce SAH. In sham-operated animals, the filament was advanced until there was resistance but no arterial puncturing was carried out. The incision was closed and rats were allowed to recover on an electric heating blanket. Buprenorphine (25 mg/kg) was subcutaneously administered immediately after surgery for pain relief. Animals had free access to food and water until euthanization.

### Experimental design

#### Experiment 1

The temporal expression profiles of TTP and PP2A after SAH were evaluated by western blotting using left cerebral cortex tissue lysates.

#### Experiment 2

SiRNAs targeting PP2A and TTP or scrambled (Scr) siRNA were administered to rats by intracerebroventricular (ICV) infusion. Behavioral testing, western blotting, and the apoptosis assay were carried out 24 h after SAH. Rats were randomly divided into five groups: sham, SAH + vehicle (normal saline, NS), SAH + Scr siRNA, SAH + PP2A siRNA, and SAH + FTY720 (PP2A agonist). Rats in the sham group were those from Experiment 1. FTY720 was administered by ICV infusion followed by siRNA treatment before SAH. Behavioral testing and western blot analysis of TTP and PP2A expression in the ipsilateral cortex were carried out 24 h after SAH.

#### Experiment 3

Rats were randomly divided into five groups: sham, SAH + vehicle, SAH + Scr siRNA, SAH + TTP siRNA, and SAH + FTY720 + TTP siRNA. Rats in the sham group were those from Experiment 1. TTP siRNA and FTY720 were administered by ICV infusion before SAH. Behavioral testing and western blot analysis of TTP expression in the ipsilateral cortex were carried out 24 h after SAH.

### ICV infusion

ICV infusion was performed as previously described (Cipriani et al., 2015; Li et al., 2016). Briefly, under 3% isoflurane anesthesia, the needle of a 10-μl syringe (Microliter #701; Hamilton Co., Reno, NV, USA) was inserted through a burr hole in the skull into the left lateral ventricle 1.5 mm posterior and 1.0 mm lateral to and 3.2 mm below the horizontal plane of bregma. FTY720 (1 μg/2 μl saline; Santa Cruz Biotechnology, Santa Cruz, CA, USA) or vehicle (NS) were injected 1.5 h before SAH induction by a pump at a rate of 0.5 μl/min. PP2A siRNA (500 pmol/3 μl; Abcam, Cambridge, MA, USA), TTP siRNA (500 pmol/3 μl; Abcam), or Scr siRNA (500 pmol/3 μl; Santa Cruz Biotechnology) were injected 24 h before SAH induction using a pump at a rate of 0.5 μl/min. In rats undergoing sham ICV infusion, a burr hole was made in the skull at the same position, but needle insertion and drug infusion were omitted. The needle was removed 5 min after completing the infusion and the burr hole was plugged.

### SAH grading

High-resolution images of the brain base (circle of Willis and basilar arteries) were acquired to assess SAH severity after euthanization as previously described (Sugawara et al., 2008). SAH severity was evaluated by an observer who was blinded to the experimental groups on a scale from 0 to 3 depending on the extent of subarachnoid blood clotting within the segment (grade 0, no subarachnoid blood in the segment; grade 1, minimal subarachnoid blood in the segment; grade 2, moderate blood clotting with recognizable arteries; and grade 3, blood clotting obliterating all arteries within the segment). Mice with SAH that was too mild (score ≤ 7 at 24 h) or too severe or that died of the injury were excluded from the groups.

### Neurological scoring

Neurological scores (3–18) were assigned before and after SAH at 24-h intervals until the time of sacrifice in all surviving animals (Garcia et al., 1995). The evaluation consisted of six tests: spontaneous activity (scored from 0 to 3), symmetry in the movement of all four limbs (scored from 0 to 3), forepaw outstretching (scored from 0 to 3), climbing (scored from 1 to 3), body proprioception (scored from 1 to 3), and response to whisker stimulation (scored from 1 to 3). The mean score of three consecutive trials at 3-min intervals was calculated, with higher scores indicating greater functioning.

### Measurement of brain water content

Brain edema was evaluated by the wet/dry method as previously described (Yan et al., 2013). Briefly, rats were anesthetized and decapitated 24 h after SAH and their brains were removed and immediately separated into the left and right cerebral hemispheres, cerebellum, and brainstem. Each part was weighted immediately after removal (wet weight) and again after drying in an oven at 105°C for 72 h. Water content was calculated according to the formula: ([wet weight] − [dry weight])/(wet weight) × 100%.

### Western blotting

Western blotting was carried out as previously described (Hu et al., 2011; Liu et al., 2014). Briefly, brains were divided into left and right cerebral hemispheres, cerebellum, and brainstem. The cerebral hemispheres opposite the blood clots were homogenized and equal amounts of protein (50 μg) were loaded on a Tris-glycine gel, separated by electrophoresis, and transferred to a nitrocellulose membrane that was blocked with blocking solution followed by overnight incubation at 4°C with the following primary antibodies: rabbit polyclonal anti-TTP (1:200), mouse polyclonal anti-PP2A (1:500), rabbit polyclonal anti-TNF-α (1:1,000), and rabbit polyclonal anti-IL-8 (1:1,000) (all from Abcam): mouse monoclonal anti-IL-6 (1:200; Santa Cruz Biotechnology); rabbit polyclonal anti-B cell lymphoma (Bcl)-2 (1:500; Sigma–Aldrich); and mouse monoclonal anti-caspase-3 (1:500; Millipore, Temecula, CA, USA). Membranes were incubated with appropriate secondary antibodies (1:2,000; Santa Cruz Biotechnology) for 1 h at 21°C, and bands were detected with a chemiluminescence reagent kit (ECL Plus; Amersham Bioscience, Arlington Heights, IL, USA). Band intensity was quantified by densitometry using ImageJ software (National Institutes of Health, Bethesda, MD, USA). β-actin (1:2,000; Santa Cruz Biotechnology) was used as a loading control.

### Terminal deoxynucleotidyl transferase dUTP nick-end labeling (TUNEL)

The TUNEL assay was carried out using the *In situ* Cell Death Detection kit (Roche, Nutley, NJ, USA) according to the manufacturer's protocol and labeled sections were analyzed with a laser scanning confocal microscope (BX51; Olympus, Shenjuku-ku, Japan). For neuronal nuclei (NeuN)/TUNEL double immunofluorescence labeling, the TUNEL reaction was performed after sections were probed with anti-NeuN primary antibody and secondary antibody. The number of TUNEL-positive neurons in five microscopic fields (400 × magnification) around the bleeding site of the subcortex was averaged for each animal.

### Statistical analysis

Data are expressed as a mean ± *SD*. Differences between groups were evaluated by one-way analysis of variance followed by the Tukey *post-hoc* test. Analyses were performed using Prism 6 software (GraphPad Inc., La Jolla, CA, USA). *P* < 0.05 were considered statistically significant.

## Results

### Mortality and SAH severity scores

No mortality was recorded in sham-operated animals and mortality rates did not differ significantly among groups (data not shown): the overall rate was 20.7%. Subarachnoid blood clots were observed around the circle of Willis 24 h after SAH. However, SAH grade scores were similar across groups (*P* > 0.05; Figure 1).

**Figure 1:** SAH grade after SAH. SAH grade following SAH (*n* = 6 per group). TTP, tristetraprolin PP2A, protein phosphatase 2A; Scr SiRNA, scrambled RNA.

### TTP and PP2A are expressed in the cerebral hemispheres after SAH

The expression of endogenous TTP and PP2A proteins in the left hemisphere (perforation side) 6, 12, 24, 48, and 72 h after SAH was evaluated by western blotting. TTP level increased after SAH and peaked at 24 h (Figure 2A; *P* < 0.05). Similarly, compared to the sham group, PP2A level increased after SAH and peaked at 24 h (Figure 2B; *P* < 0.05).

**Figure 2:** Time course of TTP and PP2A expression after SAH. **(A,B)** TTP and PP2A expression in the left cortex 72 h after SAH. Quantitative analysis of TTP and PP2A expression. (*n* = 6 per group). ^*^P < 0.05 vs. sham.

### PP2A activation suppresses neuronal apoptosis after SAH

Numerous TUNEL-positive cells were observed in the SAH as compared to the sham group, corresponding to a higher apoptotic index (*P* < 0.05; Figure 3). The apoptotic index was higher in the TTP and PP2A siRNA groups than in the vehicle groups (*P* < 0.05; Figure 3B). Treatment with the PP2A agonist FTY720 suppressed neuronal apoptosis, relative to the PP2A siRNA and TTP siRNA groups respectively (both *P* < 0.05; Figure 3B).

**Figure 3:** Effects of PP2A and TTP knockdown and FTY720 treatment on neuronal apoptosis 24 h after SAH. **(A)** Representative TUNEL (green) and DAPI staining (blue) of the left ipsilateral cortex in the indicated groups. **(B)** Quantitative analysis of TUNEL-positive neurons. The number was higher in the PP2A group and TTP siRNA groups 24 h after SAH; FTY720 decreased the number of positive neurons. Data are expressed as percentage of total cells (*n* = 6 per group). Scale bar = 50 μm. ^*^P < 0.05 vs. sham. ^#^*P* < 0.05 vs. SAH + vehicle; ^&^*P* < 0.05 vs. SAH + FTY720.

### PP2A activation reduces brain edema and improves neurological function

Brain water content was markedly elevated following SAH relative to the sham group (*P* < 0.05; Figure 4A); however, PP2A silencing increased brain water content in rats relative to those treated with vehicle (*P* < 0.05; Figure 4A). In contrast, FTY720 treatment decreased brain water content relative to the SAH + vehicle group (*P* < 0.05; Figure 4A). Neurological scores were higher in the left hemisphere of the vehicle group as compared to sham animals at 24 h (*P* < 0.05; Figure 4B). PP2A knockdown exacerbated neurological deficits associated with SAH relative to vehicle-treated rats (*P* < 0.05; Figure 4B), whereas FTY720 treatment had the opposite effect (*P* < 0.05; Figure 4B).

**Figure 4:** Expression of signaling pathway components downstream of PP2A/TTP after SAH. **(A,B)** PP2A knockdown decreased Garcia test score and increased brain water content 24 h after SAH; these effects were reversed by FTY720. **(C)** PP2A knockdown abrogated the effects of FTY720 on TTP and Bcl-2 expression and increased the levels of TNF-α, IL-6, and IL-8, and caspase-3 in the ipsilateral cortex 24 h after SAH. Relative intensity of each protein band was normalized to that in the sham group (*n* = 6 per group). ^*^P < 0.05 vs. sham; ^#^*P* < 0.05 vs. SAH+vehicle and SAH + siRNA; ^&^*P* < 0.05 vs. SAH + FTY720.

### PP2A activation reduces pro-inflammatory cytokine expression after SAH

PP2A siRNA decreased TTP expression in the ipsilateral cortex 24 h after SAH (*P* < 0.05; Figure 4C). PP2A siRNA pretreatment increased the levels of TNF-α, IL-6, and −8, and caspase-3 and decreased that of Bcl-2 (*P* < 0.05; Figure 4C). FTY720 treatment had the opposite effects (*P* < 0.05; Figure 4C).

### TTP inhibition exacerbates brain edema and neurological deficits, which is partly rescued by PP2A activation

TTP knockdown increased brain water content induced by SAH relative to vehicle-treated rats (*P* < 0.05; Figure 5A), and pretreatment with FTY720 exacerbated this effect (*P* < 0.05; Figure 5A). Neurological scores were lower in the vehicle as compared to the sham group 24 h after SAH (*P* < 0.05; Figure 5B). TTP knockdown decreased neurological function following SAH relative to animals treated with vehicle (*P* < 0.05; Figure 5B). However, these deficits were partly abrogated by FTY720 pretreatment in the TTP siRNA group (*P* < 0.05; Figure 5B).

**Figure 5:** Expression of signaling pathway components downstream of TTP after TTP knockdown and FTY720 treatment 24 h after SAH. **(A,B)** TTP knockdown decreased Garcia test score and increased brain water content in the ipsilateral cortex 24 h after SAH; these effects were reversed by FTY720 treatment. **(C)** TTP knockdown abrogated the effects of FTY720 on Bcl-2 expression and increased the levels of TNF-α, IL-6 and IL-8, and caspase-3 in the ipsilateral cortex 24 h after SAH. Relative intensity of each protein band was normalized to that in the sham group (*n* = 6 per group). ^*^P < 0.05 vs. sham. ^#^*P* < 0.05 vs. SAH + vehicle and SAH + siRNA; ^&^*P* < 0.05 vs. SAH + TTP siRNA.

### TTP inhibition increases pro-inflammatory cytokine expression following SAH

SiRNA-mediated TTP knockdown reduced TTP expression level relative to the vehicle and scrambled siRNA groups 24 h after SAH, as determined by western blotting (*P* < 0.05; Figure 5C). This was accompanied by increased TNF-α activation and IL-6 and −8 and caspase-3 expression and decreased Bcl-2 level (*P* < 0.05; Figure 5C). FTY720 treatment partly abolished these effects as compared to the TTP siRNA group (*P* < 0.05; Figure 5C).

## Discussion

Innate immune responses and inflammation contribute to the pathophysiology of EBI following SAH (Xie et al., 2017). In this study, we investigated the role of PP2A and TTP in EBI after SAH and found that silencing PP2A or TTP exacerbated brain edema and reduced neurological scores following SAH. PP2A and TTP knockdown also abolished the beneficial effects of TTP in mitigating EBI by suppressing the expression of TNF-α and IL-6 and IL-8 in the cortex. Additionally, TTP silencing reversed the anti-inflammatory effects of FTY720 *in vivo*, indicating that PP2A is associated with TTP activation and improves neurological outcome by reducing brain edema following SAH by suppressing inflammation.

TTP is an mRNA-binding protein that regulates inflammation, apoptosis, tumorigenesis, morphogenesis, and tissue development (Sanduja et al., 2012; Pandiri et al., 2016). The anti-inflammatory and anti-apoptotic effects of TTP have been reported in heart stroke, glioma (Suswam et al., 2008; Suresh Babu et al., 2015). Unphosphorylated TTP was found to induce the degradation of inflammatory mediators such as TNF-α; IL-2, IL-6, and IL-8; chemokine (C-C motif) ligand-2 and CC-3; inducible nitric oxide synthase; and other chemokines (Joe et al., 2015). PP2A dephosphorylates TTP, this interaction promotes the anti-inflammatory and anti-apoptotic functions of TTP. Our observations that inflammation and neuronal apoptosis were decreased by TTP and that these effects were enhanced by PP2A support these findings. TTP enhances the stability of ARE-containing transcripts, thereby suppressing their translation and rapid degradation (Sandler and Stoecklin, 2008). PP2A was shown to prevent inflammation-induced apoptosis in the central nervous system, lung and breast through various signaling pathways (Janghorban et al., 2014; Cheng et al., 2015; Joe et al., 2015). In the present study, TTP level was upregulated 24 h after SAH and reduced the levels of pro-inflammatory cytokines, an effect that was enhanced by PP2A activation with FTY720. This treatment also increased Bcl-2 expression and decreased that of TNF-α, IL-6, and IL-8, and caspase-3, and reduced the number of TUNEL-positive neurons while improving neurological outcome. Conversely, TTP silencing increased neuronal apoptosis and aggravated neurological deficits after SAH.

PP2A is a serine/threonine phosphatase that negatively regulates inflammation, signal transduction, cell growth, and apoptosis to protect against cardiovascular dysfunction, stroke-associated brain damage, and neurodegeneration (Shanley et al., 2001; Nematullah et al., 2017). Many studies have shown that PP2A activates TTP and is modulated by TTP activation, which suppresses inflammation in models of rheumatoid arthritis and other diseases (Mahtani et al., 2001). We showed here that PP2A and TTP knockdown induced TNF-α and IL-6 and IL-8 expression, thereby exacerbating cerebral edema and neurological impairment caused by SAH. TTP silencing abrogated the anti-inflammatory and anti-apoptotic effects of FTY720 treatment. This is consistent with a previous finding that TTP inhibited TNF-α-induced cytokine production in airway inflammation (Rahman et al., 2016). In addition to suppressing inflammation and apoptosis in a rat SAH model. Thus, PP2A-dependent TTP activation provides neuroprotection from EBI and is therefore a promising therapeutic strategy for improving neurological outcomes after SAH.

There were several limitations to this study. Many studies have proposed mechanisms to explain the anti-inflammatory effects of PP2A/TTP, including p38 MAPK phosphorylation. We cannot exclude the possibility that this plays a role in the neuroprotective effects of PP2A and TTP.

In conclusion, our results demonstrate for the first time that the anti-inflammatory and anti-apoptotic effects of TTP reduce EBI following SAH. These findings provide a basis for developing effective therapeutic strategies to improve the functional outcome of SAH patients.

## Author contributions

JY: performed the studies and wrote the manuscript; RL and WL: participated in making experimental model; YC: contributed to the TNNEL staining; XZ and XL: analyzed the sample and data; CD and XH: contributed to the design and analysis of the study and wrote the manuscript. All authors analyzed the results and approved the final version of the manuscript.

### Conflict of interest statement

The authors declare that the research was conducted in the absence of any commercial or financial relationships that could be construed as a potential conflict of interest.
